RETRACTED

# Tempol Treatment Reduces Anxiety-Like Behaviors Induced by Multiple Anxiogenic Drugs in Rats

**DOI:** 10.1371/journal.pone.0117498

**Published:** 2015-03-20

**Authors:** Gaurav Patki, Ankita Salvi, Hesong Liu, Fatin Atrooz, Isam Alkadhi, Matthew Kelly, Samina Salim

**Affiliations:** Department of Pharmacological and Pharmaceutical Sciences, College of Pharmacy, University of Houston, Houston, TX, 77204, United States of America; Technion - Israel Institute of Technology, ISRAEL

## Abstract

We have published that pharmacological induction of oxidative stress (OS) causes anxiety-like behavior in rats. Using animal models, we also have established that psychological stress induces OS and leads to anxiety-like behaviors. All evidence points towards the causal role of OS in anxiety-like behaviors. To fully ascertain the role of OS in anxiety-like behaviors, it is reasonable to test whether the pro-anxiety effects of anxiogenic drugs caffeine or N-methyl-beta-carboline-3-carboxamide (FG-7142) can be mitigated using agents that minimize OS. In this study, osmotic pumps were either filled with antioxidant tempol or saline. The pumps were attached to the catheter leading to the brain cannula and inserted into the subcutaneous pocket in the back pocket of the rat. Continuous i.c.v. infusion of saline or tempol in the lateral ventricle of the brain (4.3mmol/day) was maintained for 1 week. Rats were intraperitoneally injected either with saline or an anxiogenic drug one at a time. Two hours later all groups were subjected to behavioral assessments. Anxiety-like behavior tests (open-field, light-dark and elevated plus maze) suggested that tempol prevented anxiogenic drug-induced anxiety-like behavior in rats. Furthermore, anxiogenic drug-induced increase in stress examined via plasma corticosterone and increased oxidative stress levels assessed via plasma 8-isoprostane were prevented with tempol treatment. Protein carbonylation assay also suggested preventive effect of tempol in the prefrontal cortex brain region of rats. Antioxidant protein expression and pro-inflammatory cytokine levels indicate compromised antioxidant defense as well as an imbalance of inflammatory response.

## Introduction

Clinical evidence suggests that oxidative metabolism affects regulation of anxiety. Several groups have proposed a link between oxidative stress and certain anxiety disorders including obsessive-compulsive disorder and panic disorder [1,2]. Most clinical studies suggest associative links between oxidative stress and anxiety but causal role of oxidative stress in anxiety is not known. Animal studies on the other hand have been more informative in clarifying role of oxidative stress in anxiety-like behaviors. Several laboratories including ours have reported that pharmacological induction of oxidative stress causes anxiety-like behaviors in rats and prevention of oxidative stress with antioxidant tempol treatment mitigates anxiety-like behaviors [3–5]. These interesting studies prompted us to examine whether behavioral outcome of pharmacological induction of oxidative stress can be mimicked in situations where oxidative stress occurs as a consequence of psychological stress. Results from separate studies have revealed that the psychological stress induced via social stress [6], single-prolonged stress [7], estrogen depletion [8] and sleep deprivation [9], induce oxidative stress and also cause anxiety-like behaviors in rats. In one model of psychological stress antioxidant treatment completely rescued anxious phenotype of ovariectomized female rats [8,10].

RETRACTED

These studies have led us to test the following postulation-*if oxidative stress inducing agents cause anxiety-like behaviors*, *then anxiety-inducing agents should cause oxidative stress*., *If agents that reduce oxidative stress can reduce anxiety-like behavior*, *then effect of anxiety-inducing drugs should be overcome using antioxidants*. In the present study, we have tested whether prior antioxidant treatment prevents anxiogenic drug-induced anxiety-like behaviors in rats. Basically, two anxiety-producing drugs namely, caffeine and FG-7142 were utilized and tempol was used as an antioxidant. These drugs are reported to elicit increased anxiety-like behaviors in rodents [11]. FG-7142 is a partial inverse agonist at the benzodiazepine allosteric site on the GABA_A_ receptor and is believed to induce anxiety-like behaviors by enhancing release of dopamine, noradrenaline, and glutamate in the cerebral cortex of rodents [12]. Caffeine is an adenosine receptor antagonist known to cause anxiety-like behaviors by increasing plasma renin activity as well as elevating plasma catecholamine levels [13]. Tempol is a piperidine nitroxide and has shown antioxidant properties in various systems both *in vitro* and *in vivo*. It is a membrane-permeable radical scavenger, a pro-survival agent [14], safe to use in animals [15] and also crosses blood brain barrier [16]. In addition to measuring the effect of antioxidant treatment on caffeine/FG-7142-induced anxiety-like behaviors in rats, we also examined the status of oxidative stress both systemically as well as within three critical brain areas considered vital for anxiety, namely hippocampus, amygdala and the prefrontal cortex [17]. Levels of corticosterone (systemic marker of psychological stress) also were examined. Protein expression levels of c-fos (a biochemical marker of anxiety), the enzymes of antioxidant defense including glyoxalase (GLO)-1, glutathione reductase (GSR)-1, manganese (Mn) superoxide dismutase (SOD) and copper-zinc (Cu/Zn) SOD, inflammatory markers and a regulator of G-protein signaling protein (RGS)-2 also were examined.

RETRACTED

## Methods and Materials

### Animals

Male Sprague Dawley rats (250–275 g) obtained from Charles River, Wilmington, MA were housed in a climate-controlled room on a 12-h light/dark cycle (lights on at 0700 h). Rats were provided with food and water *ad libitum*.

### Ethics Statement

All experiments were conducted in accordance with the NIH guidelines using protocols approved from the University of Houston Animal Care and Use Committee.

### Osmotic pump implantation

One day before implantation, osmotic pumps were primed as follows: the pumps were filled with tempol (dissolved in saline; 4.3mmol/day) or saline, attached by catheter tubing to an L-shaped cannula and left overnight in isotonic saline solution at 37°C. The rats were anesthetized with i.p. injections of a mixture of ketamine (100 mg/kg; Ketaset, Fort Dodge animal health, IA), xylazine (2.5 mg/kg; Xyla-Jet, Phoenix Pharmaceuticals Inc, MO). Once anesthetized, the skin over the implantation site was shaved, cleaned with alcohol and the rat was placed on a stereotaxic frame. Starting slightly behind the eyes, a 2.5 cm midline sagittal incision was made to expose the skull. To insert the cannula, a hole was drilled into the skull (AP: -0.3, L: 1.2, V: 4.0), above the right lateral ventricle, according to the atlas of Paxinos and Watson [18]. The brain infusion cannula for saline/tempol administration was placed into the hole and held in place with instant adhesive (Locite 454, Locite corporation, CT). The osmotic pump, which was attached to the catheter leading to the brain cannula was inserted into a subcutaneous back pocket of the rat. The scalp wound was closed with wound clips and tincture of iodine, followed by triple antibiotic ointment (North safety products, RI), was applied to the wound site to prevent bacterial infection. Continuous i.c.v. infusion of saline or tempol (Santa Cruz biotechnology Inc, CA; 4.3mmol/day) was maintained for 1 week by attachment of the infusion cannula to an osmotic pump (Fig. 2).

**Fig 1:** A schematic representation of the experimental regimen. After acclimatization osmotic pumps were used to release tempol/saline by i.c.v. for 7 days. Following this rats were injected with the anxiogenic drugs or saline. Behavioral tests were performed 90 min post injection. Rats were euthanized after the behavioral tests and blood and brains harvested for future analysis.

RETRACTED

**Fig 2:** Osmotic pump release site. (A) One day before implantation, osmotic pumps were primed at 37°C. Briefly, the rats were and placed on the stereotaxic frame. A midline sagittal incision was made and a hole was drilled into the skull above the right lateral ventricle [18]. The brain infusion cannula for saline/tempol administration was placed into the hole. The pump, was inserted into a subcutaneous back pocket of the rat. (B) To confirm the site of release fast green dye was loaded into the osmotic pump, a sagittal section of the rat brain showing release site of fast green dye into the lateral ventricle of the brain.

### Drugs

On test days, rats were injected i.p. with either saline, or the adenosine receptor antagonist caffeine (Sigma-Aldrich, St. Louis, MO; 50 mg/kg) or the partial inverse agonist at the benzodiazepine allosteric site on the GABA_A_ receptor, FG-7142 (Sigma-Aldrich, St. Louis, MO; 7.5 mg/kg). Both caffeine and FG-7142 have been shown to be anxiogenic in rodents: caffeine, 50 mg/kg [19–22] and FG-7142, 7.5 mg/kg [22,23]. FG-7142 was dissolved in (40%w/v) 2-hydroxypropyl cyclodextrin (Sigma-Aldrich, St. Louis, MO) in 0.05N HCl to increase its solubility as done in previous studies [24,25]. Each of these drugs (caffeine and FG-7142) have been reported to cause increased vigilance and arousal behaviors in home cage environment of rats from when compared to vehicle-injected controls [25,26].

### Experimental design

Male Sprague Dawley rats were assigned into 6 groups; 1) Saline alone, 2) Tempol alone, 3) caffeine alone, 4) FG-7142 alone, 5) Tempol + caffeine, 6) Tempol + FG-7142. Rats in groups 1, 3 and 4 were implanted with mini-osmotic pumps containing saline and rats in groups 2, 5 and 6 were implanted with mini-osmotic pumps containing tempol. After 1 week of continuous i.c.v. infusion of saline or tempol, rats in groups 3 and 5 were i.p. injected with caffeine (50mg/kg) and rats in groups 4 and 6 were i.p. injected with FG-7142 (7.5 mg/kg). Rats in groups 1 and 2 were i.p. injected with saline. Two hours following drug injection all groups were subjected to behavioral assessments (Fig. 1).

### Anxiety-like behavior tests

First, open-field test was conducted followed by elevated-plus maze (EPM) test, 60 min after anxiogenic drug administration using our previously published behavior assays [9,27].

#### Open Field (OF) activity

Rats were placed in the center of the OF (60x40 cm) and left free to explore the arena for 15 min. Movement was quantified using a Opto-Varimax Micro Activity Meter v2.00 system (Optomax, Columbus Instruments; OH) as previously published by us [9,27]. Ambient light intensity was adjusted at 300 lux. Total activity, ambulatory activity and distance covered were determined. Ambulatory activity is the horizontal activity of the rat in the open field arena, while total activity is a combined measure of ambulatory activity and vertical activity including rearing, climbing, etc.

RETRACTED

#### Elevated plus-maze (EPM)

A standard rat elevated plus-maze with 43 cm arms extending from a 10 cm central area was used (Med Associates Inc., St. Albans, VT). The arms of the maze were approximately 90 cm above the floor. The rat’s movements were tracked visually. The observer was blinded to group classification to avoid bias. Each session which lasted 5 min was initiated by placing the rat in the central area facing the open arms of the maze. In between each test animal, the maze was wiped down with alcohol. The amount of time the rat spent in the open arms was determined [8,10,28].

### Indices of oxidative stress

8-isoprostane levels in serum were measured using EIA kit (Cayman chemical company # 516351, Ann Arbor, MI). Isoprostanes are a family of eicosanoids of non-enzymatic origin produced by the random oxidation of tissue phospholipids by oxygen radicals [27]. The OxyBlot Protein Oxidation Detection Kit (EMD Millipore Corp. # S7150) was used for immunoblot detection of carbonyl groups introduced into proteins by oxidative reactions. Equal amount (4 μg) of protein homogenate from different brain regions prepared using our published protocol [8] were subjected to this kit based reaction following manufacturer’s instructions, which allows detection of carbonylation of proteins in the homogenates using western blotting method [29].

### Plasma corticosterone

Corticosterone level in plasma was measured using an EIA based kit as previously published by us [30].

### Brain Dissections and Preparation of Homogenates

Rats were anesthetized (Isoflurane, # 57319–479–06, Phoenix Pharmaceuticals) immediately after behavior tests. The brains were quickly removed and hippocampus, amygdala and cerebral prefrontal cortex were identified according to Paxinos and Watson [18] and grossly dissected out and rapidly frozen and stored at -80°C. The isolated brain regions were homogenized and prepared as previously published by us [9]. Blood was collected and plasma was separated immediately and stored at -80°C.

### Western Blot Analysis

Equal amounts of brain tissue homogenate proteins diluted with 2X laemmli sample buffer were subjected to SDS-polyacrylamide gel electrophoresis (PAGE) and western blotting as previously published by us [9]. Primary antibody dilutions used were as follows; GLO-1 (1:200 dilution; Abcam, Cambridge, MA—Cat No: ab81461), GSR-1 (1:100 dilution), Cu/Zn SOD (1:1000 dilution; Cat No: 07–403) and Mn SOD (1:1000 dilution; Cat No: 06–984) were purchased from Millipore, Temecula, CA. c-fos (1:500 dilution; Cat No: ab184666), TNF-alpha [MP6-XT3] (1:1000 dilution; Cat No: ab11564) were purchased from Abcam, Cambridge, MA, IL-6 (1:1000 dilution; Cat No: ARC0062) was purchased from Life Technologies, Grand Island, NY. RGS-2 [N1C3–3] (1:1000 dilution; MyBiosource Inc., San Diego, CA—Cat No: MBS272204) and β-actin (1:1000 dilution; Cat No: sc-47778) were from Santa Cruz biotechnology, Santa Cruz, CA. The membranes were incubated with respective antibody for 1 h, followed by incubation with an anti-rabbit horseradish peroxidase (HRP)-conjugated secondary antibody (1:1000), anti-rat horseradish peroxidase (HRP)-conjugated secondary antibody (1:1000) or anti-mouse HRP-linked secondary antibody (1:1000) at room temperature for 1 h. The images of immunoblots were captured by a Fluorchem 8900 imaging system with intensity of each immunoreactive band determined using Alpha Ease FC 4.0 (Alpha Innotech Corp., San Leandro, CA) that were normalized to β-actin protein loading control.

RETRACTED

### Statistical Methods and Data Analysis

Data are expressed as mean ± SEM. Significance was determined by one way ANOVA followed by Tukey’s post hoc test (GraphPad software, Inc. San Diego, CA). A value of p<0.05 was considered significant.

## Results

The time spent in each compartment of the light-dark box test apparatus during 5 min test session is a reflection of aversion. Saline and tempol alone rats spent more time (sec) in the light compartment (SALINE: 86.5 ± 13.9, T: 80.0 ± 8.1), when compared to anxiogenic drugs injected rats (CAFFEINE: 31.4 ± 9.4, FG-7142: 17.1 ± 6.2) and tempol infusion prior to drug administration significantly increased the amount of time spent in the light compartment (T+CAFFEINE: 52.5 ± 7.1, T+FG-7142: 73.8 ± 14.8, *F*(5,33) = 7.41, p<0.05) (Fig. 3A). More time spent in the closed arms of the elevated-plus maze (EPM) test apparatus during a 5 min test session is indicative of high anxiety-like behavior. Saline and tempol alone rats spent more time (sec) in the open arms of the EPM (SALINE: 98.6 ± 6.8, T: 99.4 ± 9.1), when compared to anxiogenic drugs injected rats (CAFFEINE: 58.5 ± 10.2, FG-7142: 24.5 ± 9.6) and tempol infusion prior to drug administration significantly increased the amount of time spent in the open arms (T+CAFFEINE: 113.7 ± 16.7, T+FG-7142: 66.5 ± 9.4, *F*(5,33) = 7.86, p<0.05) (Fig. 3B). The open field test is frequently used as a qualitative and quantitative measure of general locomotor activity as well as of anxiety-like behavior (ref). Anxiogenic drugs injected (implanted with osmotic pump containing only saline) rats had lower total (SALINE: 4201 ± 232, T: 4112 ± 119, CAFFEINE: 2189 ± 231, FG-7142: 2494 ± 268, T+CAFFEINE: 3279 ± 300, T+FG-7142: 3551 ± 336, *F*(5,33) = 10.72, p<0.05) (Fig. 4A) and ambulatory activity (SALINE: 3563 ± 175, T: 3488 ± 121, CAFFEINE: 1827 ± 218, FG-7142: 2043 ± 212, T+CAFFEINE: 2944 ± 245, T+FG-7142: 2793 ± 288, *F*(5,33) = 11.96, p<0.05) (Fig. 4B) and covered less distance (SALINE: 3455 ± 196, T: 3405 ± 117, CAFFEINE: 1944 ± 190, FG-7142: 2091 ± 194, T+CAFFEINE: 3039 ± 317, T+FG-7142: 2772 ± 171, *F*(5,33) = 10.02, p<0.05) (Fig. 4C) than the control (saline and tempol alone) and T+CAFFEINE/FG-7142 rats. Moreover, number of fecal boli was significantly higher in anxiogenic drug injected (implanted with osmotic pump containing only saline) rats when compared to controls or T+CAFFEINE/FG-7142 (SALINE: 2.33 ± 0.6, T: 1.6 ± 0.3, CAFFEINE: 7.4 ± 1.1, FG-7142: 7.4 ± 1.2, T+CAFFEINE: 3.1 ± 0.5, T+FG-7142: 3.5 ± 1.2, *F*(5,33) = 4.79, p<0.05) (Fig. 4D). Plasma corticosterone levels were significantly increased in anxiogenic drug injected rats (CAFFEINE: 77.7 ± 3.1, FG-7142: 71.7 ± 1.8) when compared to control (SALINE: 53.8 ± 7.9, T: 40.1 ± 3.6) rats. Interestingly, rats undergoing tempol infusion prior to drug administration (T+CAFFEINE: 49.5 ± 1.8, T+FG-7142: 52.6 ± 2.1, *F*(5,26) = 24., p<0.05) (Fig. 5) had significantly lower plasma corticosterone levels when compared to CAFFEINE or FG-7142 rats.

RETRACTED

**Fig 3:** Examination of anxiety-like behavior using light-dark and elevated plus maze tests: (A) light dark and (B) elevated plus maze tests were conducted in all rats. (*) significantly different at p<0.05. Bars represent means ± S.E.M, n = 6–8 rats/group.

**Fig 4:** Examination of anxiety-like behaviors using open-field test: The open field test determined total (A), ambulatory (B) activities, distance traveled (C) and fecal boli (D) in rats. (*) significantly different at p<0.05. Bars represent means ± S.E.M, n = 6–8 rats/group.

**Fig 5:** Effect of anxiogenic drugs on plasma corticosterone levels. Anxiogenic drugs significantly elevated the plasma corticosterone levels, while tempol prevented this increase as measured using a commercially available ELISA kit. (*) significantly different at p<0.05. Bars represent means ± S.E.M, n = 6–8 rats/group.

Protein carbonylation was measured in pre-frontal cortex, amygdala and the hippocampus, brain areas, considered susceptible to oxidative stress and previously reported to be important for anxiety-like behaviors [8]. Protein carbonylation levels were not altered in the hippocampus and amygdala but significantly increased in the prefrontal cortex of the rats injected with FG-7142, while caffeine injected rats did not show an increase in protein carbonylation when compared to controls (Fig. 6A-C). Another marker of oxidative stress, plasma 8-isoprostane significantly increased in anxiogenic drugs injected (implanted with osmotic pump containing only saline) rats when compared to the controls and T+CAFFEINE and T+FG-7142 (SALINE: 12.2 ± 0.7, T: 14.9 ± 0.5, CAFFEINE: 24.6 ± 0.9, FG-7142: 23.9 ± 0.7, T+CAFFEINE: 18.0 ± 1.6, T+FG-7142: 18.7 ± 0.6, *F*(5,26) = 16.09, p<0.05) (Fig. 6D).

RETRACTED

**Fig 6:** Analysis of markers of oxidative stress. Protein carbonylation was measured using OxyBlot protein oxidation detection kit following manufacturer’s instructions (A-C). The plasma 8-isoprostane levels (D) were measured by using a commercially available ELISA kit. (*) significantly different at p<0.05. Bars represent means ± S.E.M, n = 6–8 rats/group.

Protein levels of antioxidant enzymes including Cu/Zn SOD (Fig. 7A-C), MnSOD (Fig. 7D-F), GLO-1 (Fig. 7G-I) and GSR-1 (Fig. 7J-L) were measured in the prefrontal cortex, hippocampus and amygdala regions of the brain. Both caffeine and FG-142 treatment significantly decreased Cu/Zn SOD expression while tempol treatment prevented drug-induced decline in Cu/Zn SOD levels only in the hippocampus. Protein expression levels remained unchanged in the pre-frontal cortex (Fig. 7A) and the amygdala (Fig. 7C). Mn SOD protein levels were unchanged in all three regions (Fig. 7 D-F). GLO-1 protein levels significantly increased in the prefrontal cortex of caffeine injected rats (Fig. 7G). No changes were noted in the hippocampus and the amygdala (Fig. 7 G-I). Interestingly, GSR-1 levels significantly increased in all three regions and for both caffeine and FG-7142 treated groups and tempol prevented this increase.

**Fig 7:** Examination of Cu-Zn SOD, Mn SOD, GLO-1 and GSR-1 protein levels in the prefrontal cortex, hippocampus and amygdala of rats. Protein levels of Cu-Zn SOD (A-C), Mn SOD (D-F), GLO-1 (G-I) and GSR-1 (J-L) were determined by western blotting. The upper panels are representative blots for Cu-Zn SOD, Mn SOD, GLO-1 and GSR-1 and the lower panels are protein loading control β-actin. Bar graphs are ratios of Cu-Zn SOD, Mn SOD, GLO-1 and GSR-1 to β-actin, respectively. (*) significantly different from control, p< 0.05. Bars represent means ± SEM, n = 3–5 rats/group.

The proinflammatory cytokines such as interleukin (IL)-6 and tumor necrosis factor (TNF)-α were also determined in these brain regions. The prefrontal cortex and hippocampus showed significant increase in the proinflammatory cytokines in the anxiogenic drug treated groups, while tempol prevented this increase. The amygdala displayed unchanged levels in these cytokines (Fig. 8A-F). Furthermore, RGS2 protein levels were significantly upregulated in the anxiogenic drug treated groups only in the hippocampus, while prefrontal cortex and amygdala remained unaffected. Tempol treatment prevented drug-induced increase in RGS2 expression (Fig. 9A-C). c-fos expression was upregulated across all three regions, while tempol treatment significantly reduced this increase (Fig. 9D-F).

RETRACTED

**Fig 8:** Analysis of inflammatory markers TNF-α and IL-6 in the prefrontal cortex, hippocampus and amygdala of rats. Protein levels of TNF-α (A-C) and IL-6 (D-F) were determined by Western blotting. The upper panels are representative blots for TNF-α and IL-6 and the lower panels are protein loading control β-actin. Bar graphs are ratios of TNF-α and IL-6 to β-actin, respectively. (*) significantly different from control, p< 0.05. Bars represent means ± SEM, n = 3–5 rats/group.

**Fig 9:** Examination of RGS-2 and c-fos protein levels in the prefrontal cortex, hippocampus and amygdala of rats. Protein levels of RGS-2 (A-C) and c-fos (D-F) were determined by western blotting. The upper panels are representative blots for RGS-2 and c-fos and the lower panels are protein loading control β-actin. Bar graphs are ratios of RGS-2 and c-fos to β-actin, respectively. (*) significantly different from control, p< 0.05. Bars represent means ± SEM, n = 3–5 rats/group.

## Discussion

In the present study, we provide evidence to suggest that pro-anxiety-effects of anxiogenic drugs caffeine and FG-7142 are prevented with antioxidant tempol treatment. Osmotic pumps releasing antioxidant tempol when implanted into the lateral ventricle of the brain, rescued drug-induced anxious phenotype of rats. Rats injected either with caffeine or FG-7142 alone displayed anxiety-like behaviors as measured by open field, light-dark and EPM tests. This is in agreement with previous evidence [21,22,31]. Interestingly, prior tempol infusion resulted in significant improvement in drug-induced anxiety-like behaviors when compared to caffeine or FG-7142 alone administered rats. These observations further strengthen our hypothesis that anxiety-like behaviors are regulated at least in part via oxidative stress mechanisms.

Elevated stress was also indicated by increased plasma corticosterone levels, a systemic marker of stress, in caffeine and FG-7142 alone injected rats. Drug-induced increase in corticosterone levels was markedly reduced with tempol treatment indicating anti-stress properties of tempol. Tempol infusion was carried out in the lateral ventricle which is in close proximity to the site of hypothalamic-pituitary-axis (HPA). This most likely allows tempol to modulate anxiety-induced activation of the HPA axis. This seems a reasonable postulation considering the studies of Kawabata et al. who reported suppression of CRF mRNA in the hypothalamus and decreased serum cortocisterone levels with antioxidant quercitin treatment [32]. These results are in agreement with the studies of Haleagrahara et al. who also have reported reduced serum corticosterone levels in rats with quercitin treatment [33]. Furthermore, stress mitigating effect of tempol was also evident from the c-fos data. It is well known that both systemic and neurogenic stressors [34] including anxiogenic drugs [25,26] result in activation of an early-gene c-fos expression in stress susceptible brain areas. In agreement with this, we observed that both anxiogenic drugs increased expression of c-fos across hippocampus, amygdala and the pre-frontal cortex (PFC). Drug-induced c-fos activation was prevented with antioxidant treatment, further supporting protective effects of tempol.

RETRACTED

Tempol functions via regulating oxidative stress levels [35] and increase in anxiety reportedly corresponds with rise in oxidative stress [36]. Therefore, oxidative stress parameters also were evaluated systemically as well as in the brain. Oxidative stress parameter plasma 8-isoprostane showed significant increase with anxiogenic drug administration, which was prevented with tempol treatment. This is expected as tempol is an antioxidant and known to prevent rise in oxidative stress [16,35]. Another marker for oxidative stress i.e. protein carbonylation was increased specifically in the PFC area of the brain of these rats. Our previous studies suggest hippocampus as an area more prone to protein carbonylation and hence more responsive to antioxidant treatment [10]. Perhaps, anxiogenic drugs elicit more pronounced biochemical effects in the PFC region rather than in other brain areas. Since oxidative stress occurs due to the imbalance between cellular production of reactive oxygen species (ROS) and the counteracting antioxidant mechanisms [37], we examined cellular levels of key enzymes of antioxidant defense. The expression of three antioxidant enzymes involved in the oxidative stress pathway and implicated in anxiety-like behaviors [6], GSR-1, GLO-1 and Cu/Zn SOD were altered with caffeine and FG-7142 treatment in specific brain areas. While caffeine and FG-7142-induced decrease in GSR-1 expression in the hippocampus, amygdala, and the PFC was prevented with tempol treatment, reduced levels of Cu/Zn SOD levels were noted only in the hippocampus, which also were replenished with tempol treatment. Levels of GLO-1 on the other hand were decreased only with caffeine treatment and normalized with tempol in the PFC but not in the hippocampus or the amygdala. Lack of effect in amygdala is particularly surprising considering its established involvement in stress and anxiety mechanisms [38]. Caffeine and FG-7142 clearly penetrate all three brain areas, although their relative availability in each area is difficult to assess with the approach used in the present study. Divergent effect of caffeine and FG-7142 on different antioxidant enzymes is quite apparent. This most likely is due to differential sensitivities of antioxidant enzymes for caffeine and FG-7142 and from variation in the active antioxidant enzymatic content in different areas of the brain. Furthermore, oxidative stress is reported to trigger neuroinflammation, and generate proinflammatory mediators, when ROS production exceeds the neutralizing effects of endogenous antioxidants [39]. Therefore, levels of proinflammatory cytokines including IL-6, and TNF-α were examined. We observed that the anxiogenic drug-induced rise in IL-6 and TNF-α was prevented with tempol treatment only in PFC and the hippocampus while these proteins remained unchanged in the amygdala. These results demonstrate anti-inflammatory properties of tempol. Finally, levels of RGS2 protein, which belongs to the family of small RGS proteins, commonly considered as GTPase accelerating proteins for heterotrimeric G protein α-subunits [40] was examined in the brain. RGS2 also is associated with G protein-independent functions including control of ion channel currents, microtubule polymerization, and protein synthesis [41–44] and is also considered as a stress-adaptive protein [42]. Furthermore, previous studies have shown that RGS2 modulates anxiety in both mice and humans [45–49] and also known to exert anxiolysis in one animal model [50]. Here, we observed that both caffeine and FG-7142 induced RGS2 expression selectively in the hippocampus which was normalized with tempol treatment. While these results support previous evidence of increased RGS2 expression with induction of oxidative stress [5], however, present data does not fit with the fact that lack of RGS2 causes anxiety [5]. Therefore, while reduction in corticosterone, c-fos, inflammation and up-regulation of antioxidant defense all matches with anxiolytic effect of tempol, but RGS2 diminishing effect of tempol does not fit. One attractive postulation is that RGS2 is a compensatory molecule which by regulating antioxidant expression [5] modulates anxiety-like behavior. While increase in RGS2 is part of this compensation, its decline by tempol is an antioxidant effect.

RETRACTED

In conclusion, this study demonstrates that anxiogenic drugs caffeine and FG-7142 induce anxiety-like behaviors in rats,. elevate body stress, increase oxidative stress and lead to neuroinflammation. This corresponds with decreased antioxidant defense and activation of compensatory protein RGS2. Direct infusion of antioxidant tempol in the brain mitigates anxiety-like behaviors of rats, diminishes heightened stress levels, limits oxidative stress and reduces neuroinflammation. Brain region specific effect of tempol is another attractive feature of this study. Studies examining biochemical pathways responsible for anxiolytic properties of tempol are currently ongoing.
